# miR-216b-5p Inhibited the Progression of Experimental Optic Neuritis via Downregulating FAS

**DOI:** 10.1155/2022/2772566

**Published:** 2022-08-11

**Authors:** Xiaoke Wang, Chi Ma, Lili Nie

**Affiliations:** ^1^Department of Neurosurgery, The Second Hospital of Jilin University, Changchun 130000, Jilin, China; ^2^Department of Neurosurgery, The First Hospital of Jilin University, Changchun 130021, Jilin, China; ^3^Department of Ophthalmology, The Second Hospital of Jilin University, Changchun 130000, Jilin, China

## Abstract

**Objective:**

Present study mainly explored the effect of miR-216b-5p on experimental optic neuritis and mechanism.

**Methods:**

Female C57BL/6 mice were utilized to establish the EAE model. miR-216b-5p expression was measured by RT-qPCR. Protein expression was evaluated via western blot. Inflammatory infiltration score was analyzed by HE staining. Visual function was assessed by measuring the OKR. Flow cytometry assay was conducted to measure the percentage of IL-17 cells. ELISA was utilized to evaluate the immune factor.

**Results:**

The EAE mouse model was successfully established. The EAE score of mice began to increase in EAE group after 11 days of MOG35-55 and CFA immunization. The degree of inflammatory cell infiltration in EAE mice was higher than that in normal mice. Compared with normal mice, the number of microglia and astrocytes was raised in EAE mice. miR-216b-5p expression was obviously declined and FAS expression was obviously raised in EAE. Compared with NC group, demyelination scores and axonal loss were markedly declined in miR-216b-5p mimic group. IL-17A concentration and the percentage of IL-17 cells were obviously declined in miR-216b-5p mimic group. FAS was predicted to be regulated by miR-216b-5p by TargetScan, and luciferase reporter assay confirmed this prediction. In addition, overexpression of FAS exacerbated experimental optic neuritis by promoting the inflammatory response and Th17 cell differentiation, and miR-216b-5p reversed this effect.

**Conclusions:**

miR-216b-5p downregulated FAS and inhibited the progression of experimental optic neuritis via promoting the inflammatory response and Th17 cell differentiation.

## 1. Introduction

Optic neuritis (ON) refers to various inflammatory lesions of the optic nerve, which is a more common optic nerve disease in young people [1]. According to the etiology, it can be divided into idiopathic optic neuritis, infectious and infection-related optic neuritis, autoimmune optic neuritis, and other optic neuritis that cannot be classified [2]. Among them, idiopathic demyelinating optic neuritis (IDON) is the most common type. Because IDON and multiple sclerosis (MS), which is the central nervous system demyelinating disease, have similar pathogenesis and pathological changes, it is widely believed that IDON is a part of MS [3]. The pathogenesis of MS or ON is not well understood. The more common view is that ON is an autoreactive CD4^+^ T cell-mediated autoimmune demyelinating disease directed against the central nervous system (CNS) antigens.

MicroRNAs are short stranded RNA molecules with the size of 19 to 25 nucleotides, which regulate target genes. miRNAs have been shown to be involved in the pathophysiological processes of many inflammatory diseases. For example, miR-155 promotes *T* helper cell differentiation and autoimmune demyelinating disease by inhibiting heat shock protein 40 genes dnaja2 and dnajb1 and participates in the pathogenesis of MS-ON [4]. Experimental autoimmune encephalomyelitis (EAE) is an autoimmune disease produced by sensitive animals to central nerve-specific antigens [5]. Because the EAE model has similar pathological and immunological characteristics with MS and ON, it is considered to be a classic animal model to study the pathogenesis and treatment strategies of demyelinating diseases [6]. The pathological features of ON are mainly demyelination. EAE is similar to ON in visual evoked potential (VEP) and axonal injury, which is a commonly used model for studying ON at home and abroad. Apoptosis of retinal ganglion cells (RGCs) exists in the course of optic neuritis, which leads to the thinning of retinal nerve fiber layer and affects the recovery of visual acuity, while the apoptosis of RGCs is related to immune inflammatory response and oxidative damage. In the immunopathogenesis of EAE, there is an imbalance in the Th1/Th2/Th17/Treg and their associated cytokines [7]. More and more studies in recent years confirm that the Th17/Treg imbalance plays an important role in the CNS demyelinating disease and in the pathogenesis of EAE [8]. Among them, Th17 cells secrete cytokines such as IL-17, IL-6, and TNF-*α*, which can lead to the destruction of the blood-brain barrier and aggravate the tissue inflammatory response [9, 10]. Th17 cell-associated cytokine expression levels were increased in the serum of MS and ON patients. Present study mainly explored the effect of miR-216b-5p on experimental optic neuritis and mechanism.

## 2. Materials and Methods

Clean-grade (SPF) healthy female C57BL/6 mice (6 weeks old and 18–20 g weight) were purchased from Hunan STA laboratory animal Co. Ltd. Mice were used in the experiment after being fed for one week. The antigen emulsion was placed in an ice box to ensure that the reagent emulsification process was always at low temperature. The emulsion was stirred with an electronic stir bar for 10 minutes in an ice bath. Each 0.2 mL of antigen emulsion contained 400 *μ*L MOG_35-55_ (GenScript, USA), 0.1 mL PBS, 0.1 mL CFA, and 800 *μ*g *Mycobacterium tuberculosis* lyophilized powder (Absin, China). After intraperitoneal injection of mice with 1% sodium pentobarbital sodium, the mice in the experimental group received 0.2 ml of PBS solution at 0 and 48 hours after immunization. Normal control mice were given an equal volume of PBS + CFA. Mice were observed and neurologically scored to understand progression daily from the day of immunization.

### 2.1. EAE Scoring Criteria

EAE scoring criteria are as follows: 0, normal; 1, full tail tension or ataxia; 2, full tail paralysis and ataxia; 3, double hind limb paralysis; 4, quadriplegia; 5, near death. The onset of more than 1 point was considered as EAE onset.

### 2.2. RT-qPCR

Total RNA was extracted using an RNA extraction kit (Thermo Fisher Scientific, USA). Eligible RNA was synthesized for cDNA using a reverse transcription kit (Thermo Fisher Scientific, USA). The obtained cDNA was used as templates, and qRT-PCR was conducted using the SYBR Green PCR Master Mix kit (DBI Bioscience, German). Relative expression levels of the target genes were analyzed by 2^−ΔΔCt^ method. The primer sequences of genes are shown in Table 1.

### 2.3. Histological Assessment

All mice were anesthetized by injection of 200 mg/kg pentobarbital sodium. The eyes and optic nerves were obtained to be fixed with 4% paraformaldehyde. The sections were stained with H&E method to measure inflammatory cell infiltration. Luxol fast blue (LFB, Sigma-Aldrich) was applied to detect demyelinated area, and Bielschowsky's silver staining kit (Leagene, China) was applied to measure axonal loss.

### 2.4. Optokinetic Response Recordings (OKRs)

Visual function was assessed by measuring the OKR using commercial software and apparatus (OptoMotry, Canada).

### 2.5. Luciferase Reporter Assay

The TargetScan website was utilized to predict the presence of similar binding sites between miR-216b-5p and FAS. WT-FAS containing miR-216b-5p binding site or MUT-FAS containing miR-216b-5p mutation site was constructed by Beyotime Biotechnology Co. Ltd. The CD4^+^ T-cells were co-transfected with miR-216b-5p mimics or negative control together with WT-FAS or MUT-FAS. Luciferase activity was detected after 48 h.

### 2.6. ELISA Assay

ELISA kits (Corning, USA) were utilized to detect the content of inflammatory factors, such as IL-6, IL17A, and TNF-*α*.

### 2.7. Flow Cytometry Assay

The spleen tissues of mice were placed in precooled RPMI-1640 complete medium containing 10% FBS and cell suspension was prepared. In short, cells were incubated with FITC-conjugated anti-rat CD4 and PE-conjugated anti-rat CD25. After being fixed and permeabilized, cells were incubated with PE-conjugated anti-mouse/rat IL-17A antibody (PeproTech, USA). Then, cells were sorted on a flow cytometer.

### 2.8. Western Blot

Total protein was extracted from samples, and protein concentration was determined by BCA kit. 40 *μ*L protein was added in SDS-PAGE glue and separated by electrophoresis, and the membrane was transferred to PVDF membrane, which was blocked in 5% skim milk powder for 2 h. Corresponding primary antibody (1 : 800, Abcam, USA) was added and incubated at 4°C overnight. Then, protein was incubated with secondary antibody (1 : 3 000, Abcam, USA) at room temperature for 2 h. Color was developed with ECL kit.

### 2.9. Statistical Analysis

Analysis was performed using SPSS 25.0 software. Comparisons between the two/three groups were performed using a *t*-test or one-way ANOVA.

## 3. Results

### 3.1. miR-216b-5p Was Downregulated and FAS Was Upregulated in EAE

The EAE score of mice began to increase in EAE group after 11 days of MOG_35-55_ and CFA immunization (Figure 1(a)). The degree of inflammatory cell infiltration in EAE mice was higher than that in normal mice (Figure 1(b)). Compared with normal mice, the number of microglia (Figure 1(c)) and astrocytes (Figure 1(d)) was raised in EAE mice. miR-216b-5p expression was obviously declined (Figure 1(e)) and FAS expression was obviously raised (Figure 1(f)) in EAE.

miR-216b-5p mimic obviously raised the expression of miR-216b-5p (Figure 2(a)). Compared with NC group, demyelination scores (Figure 2(b)) and axonal loss (Figure 2(c)) were markedly declined in miR-216b-5p mimic group. IL-17A concentration was obviously declined in miR-216b-5p mimic group (Figure 2(d)). The percentage of IL-17 cells was markedly decreased in miR-216b-5p mimic group (Figure 2(e)).

### 3.2. FAS Was Regulated by miR-216b-5p

FAS was predicted to be regulated by miR-216b-5p by TargetScan (Figure 3(a)). miR-216b-5p mimic obviously decreased luciferase activity of FAS-WT while it did not change luciferase activity of FAS-MUT (Figure 3(b)). In addition, FAS expression was markedly declined in miR-216b-5p mimic group (Figure 3(c)).

FAS expression was obviously raised in FAS group, and miR-216b-5p mimic markedly decreased FAS expression (Figure 4(a)). Overexpression of FAS obviously raised demyelination scores, and miR-216b-5p reversed this effect in EAE mice (Figure 4(b)). Overexpression of FAS obviously raised axonal loss, and miR-216b-5p reversed this effect in EAE mice (Figure 4(c)). Overexpression of FAS obviously raised inflammatory factor concentration, including IL-17A (Figure 4(d)), IL-6 (Figure 4(e)), and TNF-*α* (Figure 4(f)), and miR-216b-5p reversed this effect in EAE mice.

As shown in Figure 5, overexpression of FAS promoted Th17 cell differentiation and miR-216b-5p reversed this effect in EAE mice.

## 4. Discussion

Optic nerve is the main transmission pathway of visual information. ON damage can be caused by craniocerebral injury, inflammation, high intraocular pressure, and tumor growth [1]. ON is also a common optic neuropathy. The pathology of ON involves optic nerve inflammatory reaction, demyelination, and optic nerve axon injury, which can eventually lead to the loss of retinal ganglion cells and visual impairment [2]. The annual incidence of ON is about 100,000 and is considered the most common optic neuropathy in young adults. A variety of diseases can cause ON, including multiple sclerosis (MS), infectious diseases, and autoimmune diseases. MicroRNAs are considered an evolutionarily conserved class of tiny non-coding RNAs, around 22 bp in length, that play essential roles in cellular life activities and are regulators of a variety of cellular physiological processes. MicroRNAs have recently been found to regulate transcription by targeting miRNA degradation or translational repression and can directly regulate protein expression required for the proper development and function of the immune system. Recent studies suggest that miRNA is involved in the pathomechanisms of ON. miR-216b-5p is involved in the regulation of proliferation and apoptosis in cancer cells [11, 12]. miR-216b-5p has important roles in both natural and specific immunity, and its overexpression can cause chronic inflammatory diseases in humans.

In this study, the EAE mouse model was successfully established. The EAE score of mice began to increase in EAE group after 11 days of MOG_35-55_ and CFA immunization. The degree of inflammatory cell infiltration in EAE mice was higher than that in normal mice. Compared with normal mice, the number of microglia and astrocytes was raised in EAE mice. In the mice model of EAE, the optic nerve showed infiltration of inflammatory cells and myelinoclasis, which are pathological features of ON [13]. Myelin sheath is protective and supportive for the axons surrounded by it, and it is an important structure to maintain the normal conduction of action potential. Therefore, the recovery of supermyelination on demyelinated axons is a major obstacle to the treatment of ON. Oligodendrocytes (OL) are the myelin-producing cells in the central nervous system [14]. ON causes thinning of the retinal nerve fiber layer and reduces the retinal ganglion cells and their axons [15]. Therefore, observing the cell quality and quantity of RGCs became the main basis for the detection of optic nerve recovery status.

miR-216b-5p expression was obviously declined and FAS expression was obviously raised in EAE. Compared with NC group, demyelination scores and axonal loss were markedly declined in miR-216b-5p mimic group. IL-17A concentration and the percentage of IL-17 cells were obviously declined in miR-216b-5p mimic group. These results demonstrated that miR-216b-5p inhibited Th17 cell differentiation and alleviated EAE.

FAS was predicted to be regulated by miR-216b-5p by TargetScan, and luciferase reporter assay confirmed this prediction. FAS can regulate the proliferation and differentiation of a variety of cells, including Th17 cells, and then participate in the occurrence and development of autoimmune diseases. Systemic lupus erythematosus (SLE) is a chronic autoimmune disease with a major unknown etiology, and its pathological processes can almost affect organs and tissues [16]. Recent studies have found that Th17 cells can cross the blood-brain barrier in the early stage of optic neuritis and induce the activation of other inflammatory cells in the central nervous system, while Th1 plays a pro-inflammatory role in the subsequent inflammatory stage. Poissonnier et al. found that binding of Fas expressed on the surface of Th17 cells to s-CD95 in SLE patients triggered a binding domain, named the calcium-inducible domain, that was not associated with the death domain and promoted the release of Ca^2+^, thereby facilitating the migration of Th17 [17]. FAS is highly expressed during early Th17 differentiation, and FAS deletion will promote Th1 differentiation and decrease Th17 cell differentiation [18]. Activation of STATI will lead to a shift in protein expression from Fas-deficient Th17 cells to Th1 cells [19]. In addition, overexpression of FAS exacerbated experimental optic neuritis by promoting the inflammatory response and Th17 cell differentiation, and miR-216b-5p reversed this effect. Th17 cells are a subset of CD4^+^ T cells that mainly secrete IL-17 [20]. Numerous experiments showed that Th17 cells and their associated cytokines were closely related to the onset of ON and the activity of the disease [21].

In conclusion, miR-216b-5p downregulated FAS and inhibited the progression of experimental optic neuritis via promoting the inflammatory response and Th17 cell differentiation.

## Figures and Tables

**Figure 1:** miR-216b-5p was downregulated and FAS was upregulated in EAE (*n* = 15). (a) EAE score was daily recorded. (b) The extent of inflammatory cell infiltration was analyzed using H&E sections of optic nerve. (c) Optic nerve microglia number was detected by Iba-1 staining. (d) Optic nerve astrocyte number was detected by GFAP staining. (e) miR-216b-5p expression was detected by RT-qPCR. (f) Protein expression was detected by western blot. ^*∗*^*P* < 0.05. miR-216b-5p inhibited Th17 cell differentiation and alleviated EAE.

**Figure 2:** miR-216b-5p inhibited Th17 cell differentiation and alleviated EAE (*n* = 15). (a) miR-216b-5p expression was detected by RT-qPCR. (b) Demyelination score was analyzed by LFB staining. (c) Axonal loss was evaluated by Bielschowsky's silver staining. (d) IL-17A concentration was measured by ELISA. (e) The percentage of IL-17 cells was determined by flow cytometry. ^*∗*^*P* < 0.05.

**Figure 3:** FAS was regulated by miR-216b-5p. (a) Predicted binding sites. (b) Luciferase reporter assay was conducted. (c) Protein expression was measured by western blot. ^*∗*^*P* < 0.05. Overexpression of FAS exacerbated the inflammatory response and optic neuritis, and miR-216b-5p reversed this effect.

**Figure 4:** Overexpression of FAS exacerbated the inflammatory response and optic neuritis, and miR-216b-5p reversed this effect (*n* = 10). (a) Protein expression was measured by western blot. (b) Demyelination score was analyzed by LFB staining. (c) Axonal loss was evaluated by Bielschowsky's silver staining. IL-17A (d), IL-6 (e), and TNF-*α* (f) concentrations were measured by ELISA. ^*∗*^*P* < 0.05. Overexpression of FAS promoted Th17 cell differentiation, and miR-216b-5p reversed this effect in EAE mice.

**Figure 5:** The percentage of IL-17 cells was determined by flow cytometry (*n* = 10). ^*∗*^*P* < 0.05.

**Table 1:** Primer sequences.

Items	Primer sequences (5′-3′)
miR-370-3p	F : GGGGAAATCTCTGCAGGCAA
	R : CAGTGCAGGGTCCGAGGT

U6	F : GCTTCGGCAGCACATATACTAAAAT
	R : CGCTTCACGAATTTGCGTGTCAT

## Data Availability

The data used to support the findings of this study are available on reasonable request from the corresponding author.
